# Antioxidant Potential of Parsley Leaf (*Petroselinum crispum*) Essential Oil on Hypothyroidism and Testicular Injury in Mice Intoxicated by Carbon Tetrachloride

**DOI:** 10.1155/2021/9989174

**Published:** 2021-08-30

**Authors:** Gehan M. Badr, Abdulmohsen I. Algefare, Manal A. Alfwuaires

**Affiliations:** ^1^Department of Zoology, Faculty of Science, Ain Shams University, Cairo, 11566, Egypt; ^2^Department of Biological Sciences, Faculty of Science, King Faisal University, P.O. Box 380, Al-Ahsa 31982, Saudi Arabia

## Abstract

The aim of the present study was to investigate the ameliorative potential of parsley (*Petroselinum crispum*) leaf essential oil (PO) against the detrimental effects of carbon tetrachloride (CCl_4_) on the thyroid gland and testes of mice. Twenty-four adult male mice were divided into four groups and treated for 4 weeks. The 1^st^ control group received 3 mL/kg olive oil intraperitoneally, twice a week followed by 0.5 mL/kg saline intragastrically daily. The 2^nd^ CCl_4_ group received CCl_4_ (3 mL/kg intraperitoneally, twice a week). The 3^rd^ PO group received PO (0.5 mL/kg intragastrically daily), while the 4^th^ CCl_4_+PO group received CCl_4_ coadministrated with PO at the aforementioned doses. CCl_4_ group recorded significant (*p* < 0.05) reduction in the activities of antioxidant enzyme catalase (CAT) and superoxide dismutase (SOD) and significant (*p* < 0.05) increase in the lipid peroxidation end product's level malondialdehyde (MDA) in the testes and thyroid glands. Meanwhile, serum levels of testosterone, follicle-stimulating hormone (FSH), luteinizing hormone (LH), and thyroid hormones (thyroid-stimulating hormone (TSH), total triiodothyronine (T3), free triiodothyronine (fT3), total thyroxine (T4), and free thyroxine (fT4)) significantly decreased. Also, histopathologically, the testicular tissue showed hypospermatogenesis within irregular-shaped seminiferous tubules with prominent edema in the interstitial spaces confirming the aforementioned biochemical alterations. Treatment with PO significantly reduced the testicular and thyroid oxidative stress (*p* < 0.05) and elevated the testosterone (73.47%), FSH (92.11%), LH (33.33%), T3 (23.47%), fT3 (39.13%), T4 (27.91%), and fT4 (75%) as compared to that of CCl_4_-treated group corresponding values. The PO GC/MS analysis indicated bioactive monoterpenes (major component is 1,3,8-mentha triene 34.48%) and phenylpropenes (major component is myristicin 21.04%). Results suggested the ameliorative effect of PO against CCl_4_-induced hypogonadism in mice by suppressing oxidative stress and maintaining thyroid gland function.

## 1. Introduction

Oxidative stress defined as disturbance in the balance between the production of free radicals and the antioxidants (enzymatic and nonenzymatic) of the body which protect their adverse alterations in lipids, proteins, and DNA and trigger diseases. That is like its great significance for the maintenance of reproductive potential and endocrine stability in testes and ovaries [1, 2]. From the oxygen-containing free radicals occurring in many disease states are hydroxyl radical, superoxide anion radical, hydrogen peroxide, oxygen singlet, hypochlorite, nitric oxide radical, and peroxynitrite radical. The source of these reactive oxygen species (ROS) derived normally through the metabolic processes or after exposure to environmental pollutants, smoking, addiction, radiation, and infections [3, 4].

Increased testicular oxidative stress leads to germ cell apoptosis and subsequently hypospermatogenesis, where oxidative stress offered testicular changes in the dynamics of the microvascular blood flow, endocrine signaling, and germ cell apoptosis and reported as a trigger in male infertility [5]. Oxidative stress in testicular tissue decreased antioxidant enzymes and increased the production of NO, H_2_O_2_, and lipid peroxidation. Also, it increased apoptosis rate, induced DNA damage in sperm cells, and drained the seminal plasma antioxidants [6–8].

In addition, hypothyroidism is a state of increased oxidative stress [9], where the thyroid hormones regulate the metabolism of hepatocytes while the liver metabolizes thyroid hormones indicating the close connection between the liver and thyroid hormones, and dysfunction of one causes a disturbance in the other [10]. It was confirmed that hyperthyroidism markedly causes alterations of the gonadotropic and prolactin axis and dramatically affects spermatic function [11]. Hyperthyroidism is associated with oxidative stress in testicles, with increased lipid peroxidation and decreased GSH level, in addition to increased mitochondrial activity and concurrent release of electrons from mitochondrial electron transport chain due to increased production of thyroxine [12].

Carbon tetrachloride (CCl_4_) compound is used as hepatotoxic and nephrotoxic in animal models and is prooxidant which induces oxidative stress resulting in damage to body tissues by generation of free radicals, trichloromethyl (•CCl3) and trichloromethylperoxy (•CCl3O2), and other metabolites produced by cytochrome P450. They initiate lipid peroxidation by attacking polyunsaturated fatty acids in membranes, responsible for cellular damage by alteration of cellular structure, and develop through multiple organ dysfunction by these free radicals [13–18]. Oxidative stress induced by carbon tetrachloride in rats increases the level of TBARS and nitrites along with decrease in reduced glutathione and various antioxidant enzymes in testis accompanied by partial degeneration of germ and Leydig cells along with deformities in spermatogenesis [19].

Parsley (*Petroselinum crispum*; family Apiaceae) is a natural food additive and a valuable medicinal plant that is regularly consumed by humans. Parsley leaf oil, an essential oil, has a flavor that resembles that of the fresh herb. It is known to exhibit antioxidant, anti-inflammatory, and antiapoptotic effects in several tissues [20]. The major components of the essential oil extracted from parsley leaves are *α*-pinene, myristicin, and apiole [21]. In addition, Simon and Quinn reported that 1,3,8-p-menthatriene, *β*-phellandrene, myristicin, apiol, and myrcene are found in this essential oil [22]. Myristicin is a major volatile aroma constituent of parsley oil with cancer chemopreventive, anti-inflammatory, and free radical scavenging effects [23, 24]. Moreover, the two isomers *α*- and *β*-pinene are well-known monoterpenes present in parsley, and many plant essential oils have antitumor, antioxidant, and anti-inflammatory effect [25]. Also, limonene protected the cells to the oxidative stress induced by exogenous H_2_O_2_ [26]. The aim of the current study was to investigate the potential protective effect of essential leaf oil of parsley (*Petroselinum crispum*) against CCl_4_-induced oxidative stress in mouse testes and thyroid glands.

## 2. Materials and Methods

### 2.1. Plant Material

The fresh aerial parts of Parsley (*Petroselinum crispum*; family Apiaceae) were collected from the local farm of El-Sharqia Governorat, Egypt, during April 2019. The leaves were scientifically identified by a taxonomist in the herbarium of the Agricultural Museum, Giza (CAIM). A voucher specimen (CAIA 16472) was deposited at the herbarium of the Botany Department, College of Science, Ain Shams University.

### 2.2. Animals

Eight-week-old, twenty-four C57BL/6 adult male mice (25~28 g) were used in this study. The mice were maintained under standard conditions (temperature of (~20-22°C) with a 12 h light/dark cycle and 40-60% humidity and were provided with standard diet and water *ad libitum*. All experimental procedures were done in accordance with the protocol prescribed by a local ethics committee (Ref. No. KFU-REC/2021-07-01).

### 2.3. Chemical and Reagents

CCl_4_ was purchased from Sigma-Aldrich (St. Louis, MO, USA). Colorimetric assay kits of catalase (CAT; Cat. No.: CA 2516), superoxide dismutase (SOD; Cat. No.: SA 2520), and malondialdehyde (MDA; Cat. No.: MD 2528) were purchased from the Bio Diagnostic company, Giza, Egypt. The enzyme-linked immunosorbent assay (ELISA) kits of testosterone (Cat. No. MBS494055), triiodothyronine (T3; Cat. No. MBS732764), free triiodothyronine (fT3; MBS760765), thyroxine (T4; Cat. No. MBS700665), and free thyroxine (fT4; Cat. No. MBS726180) were purchased from My-Bio Source Company, San Diego, CA, USA. Thyroid-stimulating hormone (TSH; Cat. No. KT-29922) ELISA kit was purchased from Kamiya Biomedical Company (Seattle, WA, USA). ELISA kits of follicle stimulating hormone (FSH; Cat. No. KA2330) and luteinizing hormone (LH; Cat. No. KA2332) were purchased from Novus Biologicals LLC (Centennial, CO, USA). All other reagents were of analytical grade.

### 2.4. Experimental Design

After 2 weeks of acclimatization, the animals were randomly divided into four groups (6 mice per group) and treated for 4 weeks as follows:

1. Control group: administered 3 mL/kg olive oil intraperitoneally, twice a week (Saturday and Wednesday), followed by intragastrically administration daily of 0.5 mL/kg saline
2. CCl_4_ group: administered intraperitoneally, 3 mL/kg CCl_4_ (30% in olive oil), twice a week (Saturday and Wednesday), dose was chosen according to previous studies [27–29]
3. PO group: administered daily intragastrically PO (0.5 mL/kg) according to Khalil et al. [21]
4. CCl_4_ + PO group: coadministrated CCl_4_ and PO at the aforementioned doses

### 2.5. Blood and Tissue Sampling

Twenty-four hours after the last treatment, the animals were anesthetized with diethyl ether and sacrificed by cutting the neck at the jugulars by a sharp razor blade. Blood was collected into clean test tubes without anticoagulants. The blood samples were then left to coagulate at (22 ± 2) °C and centrifuged at 2800 xg for 10 min. Serum was separated immediately and stored at -80°C for future hormonal assays. Pieces of the thyroid glands and right testes were isolated and washed in ice-cold normal saline solution and kept at -80°C for future analysis. Left testes were also isolated for the histological examination.

### 2.6. Methodology

#### 2.6.1. Isolation of *Petroselinum crispum* Leaf Essential Oils

*Petroselinum crispum* leaves (700 g) were hydrodistilled in a cleveger-type apparatus [30]. After 4 h of hydrodistillation, the essential oils were recovered from water surface. The oils were then allowed to dry above anhydrous sodium sulphate and then stored in sealed dark glass vials and stored in refrigerator for additional experiments. GC-MS analysis was done by Hewlett-Packard 6890 gas chromatograph close fitting with a fused silica HP-5MS capillary column (30 m × 0.25 mm; film thickness 0.25 *μ*m). The temperature of oven was adjusted at 60°C at 3°C/min. Carrier gas was helium which was used at 2 mL/min flow rate. The gas chromatograph was coupled with a Hewlett-Packard 6890 mass selective detector. The MS working parameters were ionization voltage, 70 eV, and ion source temperature 200°C. Characterization and identification of essential oil constituents depend on their retention indices relative to n-alkanes and computer matching with the WILEY 275 Library and by comparison of the patterns of fragmentation of the mass spectra with those documented in the previous literature [31].

#### 2.6.2. Assessment of Tissue Catalase and Superoxide Dismutase Activities and Malondialdehyde Levels

The thyroid gland and testis tissues were homogenized in 0.1 M phosphate buffer. The homogenates were centrifuged at 2800 xg and 4°C for 30 min, and the supernatants were used for biochemical estimations. Catalase assay depends on the quantity of remaining hydrogen peroxide (H_2_O_2_) after the action of CAT present in the sample. The rest of H_2_O_2_ reacts with 3,5-dichloro-2-hydroxybenzene sulfonic acid and 4-aminophenazone to form colored chromophore which can be measured at 510 nm. The color intensity is inversely proportional to the amount of catalase in the original sample [32]. SOD assay relies on the ability of the enzyme to inhibit the phenazine methosulphate-mediated reduction of nitroblue tetrazolium dye that was measured at 560 nm [33]. The principal of MDA assay is thiobarbituric acid (TBA) which reacts with MDA in acidic medium at temperature of 95°C for 30 min to form thiobarbituric acid reactive product, and the absorbance of the resultant pink product can be measured at 534 nm [34]. The protein content of the tissue samples was determined by the method described by Lowry et al. using bovine serum albumin as a standard [35].

#### 2.6.3. Assessment of Thyroid Hormones in Serum

T3 ELISA kit utilized a polyclonal anti-T3 antibody and T3-HRP conjugate (T3-Horseradish Peroxidase Conjugate). The assay sample and buffer were incubated together with T3-HRP conjugate in precoated plate for one hour. Then, wells were decanted and washed five times and were incubated with a substrate for HRP enzyme. The reaction was stopped by stop solution addition to the formed blue colored complex which turned the solution yellow. The color intensity was measured spectrophotometrically at 450 nm in a microplate reader, and the T3 concentration in each sample is interpolated from this standard curve. The fT3 assay used competitive ELISA as the method where the microtiter plate provided was precoated with fT3. The sample or standard competes with a fixed amount of fT3 on the solid phase supporter for sites on the biotinylated antibody specific to fT3, and the excess conjugate and unbound sample or standard were washed from the plate. Then, HRP-Streptavidin (SABC) was added to each microplate well and incubated for 30 minutes at 37°C. Then, a TMB (3,3′,5,5′-tetramethylbenzidine) substrate solution was added to each well for about 20 minutes at 37°C. The reaction stopped by the addition of a sulphuric acid solution, and the color change is measured spectrophotometrically at a wavelength of 450 nm. The concentration of fT3 in the samples was determined as compared to the optical density of the samples to the known concentration of the standard curve. As regards the T4 assay, ELISA kit used microtiter plate precoated with an antibody specific to T4 where standards or samples were added to the plate wells with biotin-conjugated T4 and incubated for one hour at 37°C then washed three times. After washing, avidin-conjugated Horseradish Peroxidase (HRP) was added to the wells and incubated for 30 minutes at 37°C. Substrate solution was added to the wells and incubated for 15 minutes at 37°C, and the color developed was stopped, and the intensity of the color is measured at a wavelength of 450 nm in opposite to the amount of T4 in the sample that calculated as regards the standard. For the FT4 assay by ELISA kit, the assay sample and buffer were incubated together with FT4-HRP conjugate in precoated plate for one hour at 37°C. After the incubation period, the wells were decanted and washed five times, then incubated with a substrate for HRP enzyme, and a blue-colored complex was formed and turned yellow by the addition of a stop solution, and the color intensity was measured spectrophotometrically at 450 nm in a microplate reader. The FT4 concentration in each sample is interpolated from the standard curve.

The TSH assay ELISA kit used antibody specific to TSH precoated microplate. A detection reagent was added to each well and was incubated for 1 hour at 37°C. After incubation, the unbound conjugate is washed off. Next, avidin conjugated to Horseradish Peroxidase (HRP) was added to each microplate well and incubated for 30 minutes at 37°C. Then, a substrate solution was added to each well and incubated for 15 minutes at 37°C, and the color developed was stopped by the addition of stop solution, and the intensity of the color is measured at a wavelength of 450 nm. Concentration was determined by using calibration curve on log-log or semilog graph paper, with the log of TSH concentration on the *y*-axis and absorbance on the *x*-axis, and the best fit straight line through the calibrator points was drawn and determined by regression analysis.

#### 2.6.4. Assessment of Testicular Hormones in Serum

Serum testosterone levels were measured using an ELISA kit. The principal is based on the competitive binding reaction between unknown hormone in our sample and known hormone sample conjugated to horseradish peroxidase (HRP). They compete for the binding sites of microplate wells coated with antitestosterone antibody. After one-hour incubation on a shaker (600 rpm), the microplate is washed four times. Then, a substrate solution is added and is incubated in dark for 30 minutes, and reaction is stopped by stop solution, and the optical density was measured spectrophotometrically at 450 nm. The concentration of testosterone (pg/mL) is calculated against reference stranded assayed in the same way.

The FSH assay is based on a solid phase enzyme-linked immunosorbent assay, where test sample is reacted with two antibodies, a rabbit polyclonal anti-rat FSH antibody for solid phase (microtiter wells) immobilization and a goat anti-rat FSH antibody in coupled to enzyme (horseradish peroxides) conjugate solution. FSH molecules were sandwiched between the solid phase and enzyme-linked antibodies for a 3-hour incubation period at 37°C, then wells are washed for unbound labeled antibody removal. A color reagent solution is added and incubated for 20 minutes, developing a blue color that is stopped by addition of 2 N HCl, and the intensity of the color formed is measured spectrophotometrically at 450 nm. The concentration (ng/mL) of LH in sample was calculated in reference to a series of FSH standards assayed in the same way. While in LH assay like in FSH assay, test sample is reacted with two antibodies, a mouse anti-LH antibody for solid phase (microtiter wells) immobilization and mouse anti-LH antibody in the antibody-enzyme (horseradish peroxidase) conjugate solution. LH molecules sandwiched between the solid phase and enzyme-linked antibodies for a 2-hour incubation, then wells are washed with wash buffer to remove unbound labeled antibodies. A color reagent solution is added and incubated for 20 minutes, developing a blue color that is stopped by addition of 2 N HCl, and the intensity of the color formed is measured spectrophotometrically at 450 nm. The concentration of LH (ng/mL) in sample was calculated in reference to a series of LH standards assayed in the same way.

#### 2.6.5. Assessment of Histological Alterations Using Light Microscopy

The testes were fixed in 10% formaldehyde solution at 28°C for 24 h, dehydrated, and embedded in paraffin wax. Thin sections were stained with conventional hematoxylin and eosin (H&E) dye. The slides were examined using a standard light microscope (Nikon Corporation, Tokyo, Japan). Johnsen's tubular biopsy score (JTBS) [36] was used to evaluate the degree of testicular damage and maturity in 20 seminiferous tubules (magnification 400x) for each sample. In this respect, a numerical score of 1–10 was assigned to each seminiferous tubule indicating level of germinal epithelial maturation as follows: score (1), atrophic tubule; score (2), Sertoli cells without germ cells; score (3), only spermatogonia can be seen and no primary spermatocytes; score (4), few primary spermatocytes; score (5), many spermatocytes; score (6), few round spermatids; score (7), large number of early spermatids without differentiation; score (8), few late spermatids; score (9), many late spermatids; and score (10), regular tubules with lots of sperm. Also, histomorphological analysis was assessed by measuring the diameter of 20 seminiferous tubules across the minor and major axes by using the imaging software (NIS-Elements, Tokyo, Japan), and the mean diameter was obtained. The tubular diameter was measured at magnification 400x. Round or nearly round tubules were randomly chosen.

### 2.7. Statistics

All data are expressed as means ± standard error (SE). Statistical calculations were performed using Graph Pad Prism (version 3.00 for windows, GraphPad software, San Diego, CA, USA) The results were analyzed by one-way analysis of variance (ANOVA) for the comparison of the differences between the experimental groups followed by Tukey's post hoc test. The statistical level of significance was set at *p* < 0.05.

## 3. Results

### 3.1. Identification of Chemical Composition of Parsley (*Petroselinum crispum*) Leaf Essential Oil

Hydrodistillation of the *Petroselinum crispum* leaves yielded 1.45% of clear yellowish liquid oil, where ten components, representing 100% of the total oil, were identified, and their percentages were calculated and are shown in Table 1 and Figure 1. The monoterpene components were 1, 3, 8-mentha triene (34.48%), *β*-pinene (5.79%), *β*-phellandrene (4.65), *α*-pinene (4.61%), myrcene (3.48%), limonene (3.23%), and terpinolene (1.75%). The phenylpropene compounds were myristicin (21.04%), apiole (18.08%), and elemicin (2.89%).

### 3.2. Antioxidant Effect of PO on Thyroid and Testicular Tissues

The results in Table 2 revealed that mice intoxicated with CCl_4_ recorded a decrease in CAT and SOD enzyme activities and a significant increase in MDA levels in comparison with the control group corresponding values. Coadministration with PO markedly decreased the toxicity of CCl_4_ by significantly increasing the enzymatic activities of CAT and SOD and significantly decreasing MDA levels toward the CCl_4_ group corresponding values. The group treated with PO alone showed not statistical differences in the detected parameters levels as compared to their corresponding control group.

### 3.3. Ameliorative Effect of PO on Thyroid Hormones

Figure 2 shows a significant decrease in T3, fT3, T4, fT4, and TSH levels in mice treated with CCl_4_ when compared to the control values. Compared to the CCl_4_ and control groups, the group administered with CCl_4_ and PO showed significant elevations and reductions in the levels of thyroid hormones, respectively. However, the thyroid hormones assayed in PO group recorded not statistical differences from their corresponding control group.

### 3.4. Modulatory Effect of PO on Testicular Hormones

Figure 3 represented the significant decrement effect of CCl_4_ administration in CCl_4_ group in the levels of testosterone, FSH, and LH. The group treated with CCl_4_ and PO showed a significant increase in these levels compared to the CCl_4_ group but showed a significant decrease when compared to the control group. The PO-treated group showed no changes when compared to the control group.

### 3.5. Protective Effect of PO on Testis Histology

Figure 4 shows the histoarchitecture (a, b, and c), histopathological scoring (d), and the histomorphological diameter of seminiferous tubules (e) of testes. The control group exhibited regular and normal seminiferous tubules and a normal spermatogenesis series (a). CCl_4_ treatment resulted in hypospermatogenesis within irregular-shaped seminiferous tubules. Further, this group showed notable germinal cell destruction compared to the control group. In addition, the testicular tissue sections exhibited desquamation and vacuolization in the germinal epithelium with prominent edema in the interstitial spaces (b). Conversely, the effects on the seminiferous tubule structure were ameliorated in the group treated with CCl4 and PO, in addition to improvement in the spermatogenesis series. However, some detachments in the seminiferous epithelium, edema, and congestion were still detected in the testicular tissues of this group (c). The mean testicular spermatogenesis scores by JTBS (d) values were compared among groups. The mean of JTBS was 3.2 in CCl_4_ group that was significantly lower than the value in control group (9.5), indicating atrophy and hypospermatogenesis, while the coadministration with PO significantly increased JTBS values (5.8) as compared to that recorded in CCl_4_ group. The results of the histomorphological seminiferous tubule diameter means (e) were compared among groups. The CCl_4_ group showed 121.4 *μ*m diameter which is significantly lower than that of control group (144.1 *μ*m), while coadministration with PO recorded significantly increased mean of tubule diameter values (136.7 *μ*m) as compared to the CCl_4_ group value.

## 4. Discussion

It is well known that CCl4 is a potent hepatotoxin and used to induce acute liver injury in experimental animal models by mechanisms involving oxidative stress, lipid peroxidation in the hepatocyte membrane, inflammatory responses, and hepatocyte apoptosis and necrosis [37]. The present study results revealed the CCl_4_ induction of the oxidative stress status through the altered cellular redox balance in both testicular and thyroid tissues. There is a recorded significant reduction of the antioxidant enzyme activities of SOD and CAT, where SOD catalyzes the dismutation of superoxide radical into oxygen and hydrogen peroxide and CAT catalyzes the decomposition of hydrogen peroxide to water and oxygen, in addition to the significant elevated levels of the lipid peroxidation marker, MDA, in the aforementioned tissues. Hence, the enhanced lipid peroxidation and reduced antioxidant enzyme activities lead to increased accumulation of superoxide radicals which additionally stimulate more lipid peroxidation. This oxidative stress status was previously confirmed through conversion of CCl4 to free radicals through cytochrome P450 enzymes that induce a chain reaction causing lipid peroxidation in the cell membrane, mitochondria, and endoplasmic reticulum, as well as membrane oxidative phosphorylation, which triggers cellular apoptosis and necrosis [38, 39]. The imbalance between the free radicals and the antioxidant defense system which induced damage in the nucleic acids, proteins, and lipids present in the sperm membrane was reviewed, where the structural integrity of the sperm membrane maintained by cholesterol and phospholipids and possesses a large quantity of polyunsaturated fatty acids that make the sperm highly vulnerable to oxidative stress. In addition the low concentrations of antioxidant enzymes like catalases and dismutases, the sperm plasma membrane leads it to be susceptible to the attack of the free radicals triggering alterations in the membrane permeability for entrance of cations into the sperm, shifting its osmolarity, and leading to formation of soluble calcium phosphates, depletion of ATP, and activation of proteolytic and phosphoglycolytic enzymes. In addition, such damages lactate dehydrogenase, pyruvate kinase, glyceraldehyde 3 phosphate dehydrogenase, and ATPase enzymes that leads to loss or decreases in sperm mobility, protein and lipid damage, DNA alterations, anomalies in its morphology, fertility problems, and cell death [40]. That is in line with the present study result consequence in the demonstrated significant decrease in testosterone, FSH, and LH levels in the CCl4 group. And the histopathological examination of the testicular tissue in CCl_4_ group revealed hypospermatogenesis (JTBS), reduced diameter of seminiferous tubules, and destructed germinal cells compared to the control group. Hypogonadism effect as a result of CCl4-induced oxidative stress may be due to the direct toxicity of CCl4 on the Leydig cell membrane and central nervous system or due to its indirect effect on the hypothalamic–pituitary–gonadal axis as previously discussed in many studies [19, 41–46].

The thyroid gland oxidative stress status and the hypothyroidism predicted by the decreased T4, T3, fT4, fT3, and TSH levels in the CCl4 group in the present study are in agreement with the thyroid gland malfunction due to CCl4 intoxication previously evaluated in different experimental studies, where CCl4 increased lipid peroxidation and decreased the level of antioxidant enzymes in thyroid tissue, and the serum levels of thyroid hormones are affected by mechanisms that interfere with the hepatic metabolism of thyroid hormones, i.e., via suppressing the activity of outer ring deiodine enzyme that converts T_4_ into the biologically active T_3_ form in liver microsomes, and CCl_4_ may directly affect pituitary–thyroid axis hormones [10, 19, 27, 47–52].

The chemical compositions of parsley oil are previously evaluated in many studies from different plant varieties and seasonal variations by different extraction methods that could affect the content percentage of the identified compounds. The main separated components in the present results were 1,3,8-mentha triene, myristicin, and apiole, that monoterpene and phenylpropene compounds are consistent with previous studies as main compounds with antioxidant activities [53–56]. The compounds making the greatest contributions to characteristic parsley odor are 1,3,8-mentha triene and apiole. Myristicin, apiole, *α*-pinene, and *β*-penene scavenge free radicals and induce antioxidant enzyme production in cells, thus protecting against ROS generated by CCl4-induction [23, 53, 55, 57, 58]. In addition, PO may stimulate the synthesis of glutathione, which is a crucial nonenzymatic antioxidant [59]. The antioxidant activity has been confirmed using the 1,1-diphenyl-2-picrylhydrazyl (DPPH) radical scavenging and *β*-carotene–linoleate bleaching assays as well as Ferric reducing capacity method [55, 60] Hence, the presence of bioactive compounds may be a key factor in reducing the free radicals, where PO coadministration with CCl4 impedes oxidation in testicular and thyroid tissues through the recorded significantly increased enzymatic activities of CAT and SOD and decreased MDA levels in the testicular and thyroid tissues as compared to CCl4 group. Antioxidant enzymes play key roles in the detoxification of free radicals and ROS produced during exposure to toxic chemicals, including the metabolism of various xenobiotics such as CCl4 [27]. Also, previous studies reported that antioxidant compounds can protect the testis tissue against apoptosis and prevention of lipid peroxidation [61, 62]. In addition, PO may stimulate the synthesis of glutathione, which is a crucial nonenzymatic antioxidant [59].

A significant improvement was observed in thyroid and testicular hormone profiles of the group coadministered with PO and CCl4 compared to that of the CCl4 group by their significant increase and evaluated through the histological improvement of the testicular tissue. In agreement with the study of Razooqi et al. [63], they reported that PO has a protective role against heat stress-induced damage to the testes of Japanese quail. Moreover, the ameliorative effect of parsley on thyroid gland dysfunction has been linked to its antioxidant effects or indirectly via its hepatoprotective effect as PO coadministration attenuated thyroid hormone metabolic disturbances associated with liver injury induced [49, 59, 64, 65]. In addition, PO was therapeutically recommended in a previous study in hypothyroidism mice model via its elevating effect on thyroid hormones and the histopathological evidenced recovery of thyroid parenchyma [64] as regards the effect of thyroid hormones on different cell types in the testes, such as the Leydig cells, Sertoli cells, and germ cells, with T3 regulating testicular growth and maturation [65]. Thyroid hormone receptors have been identified in the testes; therefore, thyroid hormones are considered to have key roles in male reproductive functions [66, 67]. In addition, Badr et al.'s study showed that testicular damage caused by cadmium in rats can be improved by reversing the hypothyroid status via treatment with quercetin, a natural antioxidant [68]. Moreover, recent study showed that natural antioxidants alleviated testicular toxicity in rats with hypothyroidism [69].

## 5. Conclusion

The present study results recommended that the natural antioxidant and parsley essential oil administration via its constituents could induce amelioration of thyroid hormone levels and improvement in the testicular injury in mice intoxicated by CCl4. Meanwhile, further studies are required for the evaluation of PO activities which missed in the present study including the evaluation of more parameters of the antioxidant system and the molecular basis of these protective and therapeutic effects in testicular tissue.

## Figures and Tables

**Figure 1:** GC-MS chromatograph of parsley (*Petroselinum crispum*) leaf essential oil.

**Figure 2:** Effect of oral administration of PO (0.5 mL/kg) on the thyroid gland hormone profile in mice intoxicated with CCl_4_; *n* = 6. (a) T3, (b) fT3, (c) T4, (d) fT4, and (e) TSH. Results are expressed as mean ± SE. Bars with different letters are significantly different (*p* < 0.05) between groups.

**Figure 3:** Effect of oral administration of PO (0.5 mL/kg) on the testicular hormone profile in mice intoxicated with CCl_4_; *n* = 6 per group. (a) Testosterone, (b) FSH, and (c) LH. Results are expressed as mean ± SE. Bars with different letters are significantly different (*p* < 0.05) between groups.

**Figure 4:** Light micrographs of testicular tissues of the experimental groups represented in (a–c). Control group (a) exhibiting regular seminiferous tubule (arrow) with normal spermatogenesis series (Sp). CCl_4_ group (b) demonstrating irregular and marked damage of seminiferous tubules, desquamation (D), edema (E), vacuolization (V), and congestion (C). CCl_4_ + PO (c) showing histological improvements. Hematoxylin and eosin staining with original magnification 400x. (d) Johnsen's tubular biopsy score (JTBS), and the histomorphological diameter of seminiferous tubules (*μ*m) were represented in (e). Bars with different letters are significantly different (*p* < 0.05) between groups.

**Table 1:** Chemical composition of parsley (*Petroselinum crispum*) leaf essential oil.

Retention time (min)	Compounds	Area %	Chemical class
25.34	1,3,8-Mentha triene	34.48	Monoterpene
25.395	Myristicin	21.04	Phenylpropene
25.530	*α*-Pinene	4.61	Monoterpene
25.578	Elemicin	2.89	Phenylpropene
25.677	Limonene	3.23	Monoterpene
25.754	*β*-Pinene	5.79	Monoterpene
26.821	Terpinolene	1.75	Monoterpene
27.832	*β*-Phellandrene	4.65	Monoterpene
28.705	Apiole	18.08	Phenylpropene
29.447	Myrcene	3.48	Monoterpene

**Table 2:** Effect of oral administration of PO (0.5 mL/kg) on thyroid and testicular tissues antioxidant parameters.

Groups	Parameter					
	CAT (U/mg protein)		SOD (U/mg protein)		MDA (nmol/g tissue)	
	Testis	Thyroid	Testis	Thyroid	Testis	Thyroid
Control	34.58 ± 0.39^a^	23.62 ± 0.76^a^	63.30 ± 0.48^a^	42.35 ± 0.54^a^	8.76 ± 0.18^a^	7.183 ± 0.18^a^
CCl_4_	15.08 ± 0.29^b^	8.833 ± 0.27^b^	20.43 ± 0.17^b^	17.98 ± 0.26^b^	31.07 ± 0.47^b^	21.02 ± 0.47^b^
PO	33.68 ± 0.39^a^	23.03 ± 0.41^a^	62.28 ± 0.50^a^	41.2 ± 0.60^a^	9.12 ± 0.34^a^	6.707 ± 0.16^a^
CCl_4_+PO	22.12 ± 0.57^c^	13.13 ± 0.48^c^	35.68 ± 0.53^c^	25.85 ± 0.22^c^	18.05 ± 0.37^c^	12.67 ± 0.39^c^

Data are expressed as mean ± SE. Different superscript letters within the same column are significantly different (*p* < 0.05).

## Data Availability

The data used to support the findings of the study are available from the corresponding author upon request.
